The article "Safety and Feasibility of Robotic Natural Orifice Specimen Extraction Surgery in Colorectal Neoplasms During the Initial Learning Curve" was published in 2020. Journal: Front Oncol.

# Safety and Feasibility of Robotic Natural Orifice Specimen Extraction Surgery in Colorectal Neoplasms During the Initial Learning Curve

**DOI:** 10.3389/fonc.2020.01355

**Published:** 2020-09-11

**Authors:** Hongliang Yao, Tiegang Li, Weidong Chen, Sanlin Lei, Kuijie Liu, Xiaoxin Jin, Jiangjiao Zhou

**Affiliations:** Department of General Surgery, The Second Xiangya Hospital, Central South University, Changsha, China

**Keywords:** colorectal neoplasms, learning curve, natural orifice specimen extraction surgery (NOSES), robotic surgery, safety and feasibility

## Abstract

**Aim:** To analyze the learning curve (LC) for robotic natural orifice specimen extraction surgery (NOSES) for colorectal neoplasms and evaluate safety and feasibility during the initial LC.

**Method:** Patients who consecutively underwent robotic NOSES performed by two surgeons between March 2016 and October 2019 were analyzed retrospectively. The operation time was evaluated using the cumulative sum method to analyze the LC. The clinicopathological data before and after the completion of LC were extracted and compared to evaluate safety and feasibility.

**Results:** In total, 99 and 66 cases were scheduled for robotic NOSES by Prof. Yao and Prof. Li, respectively. The peak points of LC were observed at the 42nd and 15th cases of Yao and Li, respectively, then operation time began to decrease. Only the operation time for Yao before the completion of LC (213.3 ± 67.0 min) was longer than that after the completion of LC (143.8 ± 33.3 min). For Yao nor for Li, other indices, such as postoperative hospital stay, intraoperative blood loss, conversion to laparotomy, incidence of anastomotic leakage, reoperation rate, and 90-day mortality rate lacked significant statistical differences(*P* > 0.05). In terms of feasibility, the number of lymph nodes harvested, positive resection margin rate, and total cost before and after the completion of LC had no significant statistical difference (*P* > 0.05).

**Conclusion:** The cases before the completion of LC for robotic NOSES in colorectal neoplasms varied from 15 cases to 42 cases. Robotic NOSES is safe and feasible during the initial LC.

## Statement

Laparoscopic NOSES is mature, but robotic NOSES should have a faster LC and some advantages. How many cases needed to complete LC of robotic NOSES? Is it safe during the initial LC? This is an analysis of LC on the world's maximum cases of robotic NOSES in colorectal neoplasms.

## Introduction

Minimally invasive surgery is the developmental tendency of colorectal surgery. After decades of development, laparoscopic colorectal surgery has become mature, and its safety and effectiveness are no less than those of open surgery. Moreover, laparoscopic surgery is with the virtue of fast recovery and minimal trauma. Although laparoscopic surgery does not require large incisions unlike open surgery, it still requires a small incision to extract specimens. This requirement leads to abdominal incision pain and wound complications, including infection, hernia formation, and scarring.

The article "Safety and Feasibility of Robotic Natural Orifice Specimen Extraction Surgery in Colorectal Neoplasms During the Initial Learning Curve" was published in 2020. Journal: Front Oncol.

NOSES is a kind of operation that can realize the “no scar” concept to the limit and uses a soft endoscope or laparoscope to enter the abdominal or chest cavity through the mouth, gastrointestinal tract, vagina, bladder, or other natural orifice to conduct medical procedures, including exploration, biopsy, appendectomy, hysterectomy, and cystectomy, without any auxiliary incision on the body surface (1). In 2007, the French doctor Marescaux has completed transvaginal cholecystectomy, the first truly scar-free operation in the world. Thus, the minimally invasive requirements of surgery have entered a new era (2).

NOSES is especially suitable for colorectal surgery. Incisions in the oral cavity, rectum, vagina, and other natural orifices must be made to remove the specimens from the natural lumen for appendectomy, cholecystectomy, and nephrotomy. For colorectal neoplasms, however, the rectum needs to be disconnected during colorectal surgery, and then the rectum and anus can act as natural orifices for specimen extraction. This approach can avoid making any artificial incision and has natural advantages.

The Da Vinci surgical robot has been approved by the FDA since 2000. Compared with laparoscopic surgery, robotic surgery is more advanced with several benefits, such as superior three-dimensional vision and EndoWrist instruments which can achieve a wide range of motion, and a shorter learning curve (LC). However, the safety and feasibility of robotic NOSES during the initial LC and the possibility for shortening the LC remain unclear. Therefore, this work addressed the LC of robotic NOSES in our hospital through a retrospective analysis. At the same time, the clinicopathological data before and after the completion of LC were compared to analyze the safety and feasibility of robotic NOSES during the initial LC.

## Methods

This work has been reported in line with the STROCSS criteria.

### Patients Selection

This is a retrospective study on robotic NOSES for patients with sigmoid and rectal neoplasms performed by two surgeons, Prof. Yao and Prof. Li. Yao and Li had performed more than 1,000 open radical resections of colorectal cancer before October 2015. In October 2015, the Da Vinci Si Robot Surgical System was installed in the hospital. All patients diagnosed with sigmoid and rectal neoplasm between March 2016 and October 2019 were confirmed for resectability before operation. The exclusion criteria for robotic NOSES were as below: (1) age <18 years old; (2) emergency operation due to gastrointestinal obstruction, perforation, or bleeding; (3) any suspicious invasion of the pelvic wall, bladder, or any other perirectal tissue or organs; (4) written informed consent of patients cannot be obtained; (5) specimen was unexpectedly removed through the anus by preoperative evaluation; (6) body mass index ≥ 28 kg/m^2^; (7) metastasis of lung, bone, or liver that cannot be removed simultaneously; and (8) patients with contraindication that cannot tolerate robotic NOSES. Given that our study focuses on the LC of robotic NOSES for patients with sigmoid and rectal neoplasms, cases combining the resection of other organs, such as ovariectomy and hysterectomy, were excluded. This work is in accordance with the declaration of Helsinki and is approved by the Ethics Committee of Hospital.

The article "Safety and Feasibility of Robotic Natural Orifice Specimen Extraction Surgery in Colorectal Neoplasms During the Initial Learning Curve" was published in 2020. Journal: Front Oncol.

### Surgical Technique

After successful general anesthesia, the patient assumed the Trendelenburg position. Five trocars were needed (one for the robotic camera, three for the robot operation arms, and one for the assistant). First, in accordance with the principle of total mesorectal resection or complete mesocolon resection, the blood vessels were ligated at the root of the inferior mesenteric artery, and the rectum or sigmoid colon and its mesentery were completely free, whereas the left ureter was protected properly. The left colonic artery was preserved. At 10 cm from the proximal and 2–5 cm from the distal of the tumor, the rectum was ligated with a self-locking nylon bandage and then amputated. After the assistant had fully dilated the anus, an endoscope sterile sleeve was placed into the pelvic cavity through the anus. One end of the sterile sleeve was kept outside the anus, and the other end was kept inside the pelvic cavity. Sponge forceps were placed into the pelvic cavity through the sterile sleeve, and the proximal end of the removed sigmoid colon or rectum was clamped and slightly dragged outward. After the specimens were all in the sterile sleeve, the inner end of the sleeve was ligated such that the specimens would not slide out from the sterile sleeve. The assistant pulled the sponge forceps to pull out the sterile sleeve and the specimens together through the anus. Then, the assistant situated the orvil of the stapler into the pelvic cavity from the anus. The operator sutured the stump of the sigmoid colon and placed the orvil in it. After the operator sutured the stump of the rectum, the assistant placed the stapler through the anus to complete the anastomosis. Then, air was pumped into the rectum via the anus to determine the presence of air leakage from the anastomosis. If air leakage or serous membrane eversion was present, additional sutures can be performed (Figure 1). The perioperative management followed international guidelines (3).

The article "Safety and Feasibility of Robotic Natural Orifice Specimen Extraction Surgery in Colorectal Neoplasms During the Initial Learning Curve" was published in 2020. Journal: Front Oncol.

**Figure 1:** Surgical procedure. **(A)** The inferior mesenteric artery and vein were isolated and clipped by absorbable vascular clamps; **(B)** Rectum was ligated with self-locking nylon bandage; **(C)** Sigmoid colon was ligated with self-locking nylon bandage; **(D)** Suture the stump of sigmoid colon and put the orvil into the sigmoid colon; **(E)** Suture the stump of rectum; **(F)** Complete the anastomosis.

### Date Collection

All perioperative data, including the following variables, were collected retrospectively for analysis.

1. General information of patients: gender, age, chief complaints, comorbidities, American Society of Anesthesiology (ASA) classification;
2. Perioperative data: operative time (OT), intraoperative blood loss, laparotomy conversion rate;
3. Postoperative data: postoperative hospital stay, pathological results, short-term complications, anastomotic leakage, 90-day mortality, reoperation rates, total medical expenses,

Pathological information was recorded on the recommendation of AJCC 8th Edition Cancer Staging Form. Postoperative complications were classified using the Clavien–Dindo classification of surgical complications (4).

### Statistical Analysis

SPSS (version 25.0, Chicago, USA) was used for analyzing. Measurement data expressed as mean ± standard deviation, and count data were presented as numbers and percentages. The measurement data and count data were statistically analyzed with two-tailed Student's *t*-test and Pearson's χ^2^ test, respectively. *P* < 0.05 was considered to demonstrate statistically significant differences.

The cumulative sum (CUSUM) technique was used to detect a shift in the trend of OT. Robotic NOSES cases were arranged in chronological order. CUSUM_OT1st_ is the difference between OT_1st_ and the mean OT, i.e., OT_1st_-OT_mean_. CUSUM_OT2nd_ is calculated as CUSUM_OT_ _1st_ + (OT_2nd_-OT_mean_). CUSUMOT _3rd_ is calculated as CUSUMOT _2nd_ + (OT_3rd_-OT_mean_). So, CUSUM_χ_ = CUSUM_χ−1_ + (OT_χ_- OT _mean_). Then notable OT change points could be observed at the peak in the CUSUM curve.

## Results

### Details of Patients and Clinicopathological Characteristics

In total, 99 and 66 cases of robotic NOSES were performed by Yao and Li, respectively, between March 2016 and October 2019. Details are provided in Table 1.

**Table 1:** Clinicopathological characteristics of all patients.

	**Prof. Yao**		**Prof. Li**		***P***
	**Cases (n)**	**Ratio (%)**	**Cases (n)**	**Ratio (%)**	
Gender					0.429
Male	60	60.6	44	66.7	
Female	39	39.4	22	33.3	
Age (mean ± SD)	57.8 ± 12.8		57.4 ± 13.2		0.864
20–39	8	8.1	7	10.6	
40–59	42	42.4	28	42.4	
60–79	44	44.4	27	40.9	
≥80	5	5.1	4	6.1	
ASA score					0.933
1	4	4	3	4.5	
2	47	47.4	34	51.5	
3	47	47.4	28	42.4	
4	1	1	1	1.5	
History of abdominal surgery					0.857
Yes	14	14.1	10	15.2	
No	85	85.9	56	84.8	
nCRT					0.076
Yes	17	17.2	5	7.6	
No	82	82.8	61	92.4	
Protective ileostomy					>0.99
Yes	4	4	2	3	
No	95	96	64	97	
Distance from the lower edge of the tumor to the anus					0.116
<5 cm	4	4	7	10.6	
5–10 cm	53	53.5	39	59.1	
≥10 cm	42	42.4	20	30.3	
CDmax					0.252
<3 cm	35	35.4	16	24.2	
3–5 cm	46	46.5	33	50	
≥5 cm	18	18.2	17	25.8	
T staging					0.023
Tis	0	0	1	1.6	
T1	7	7.4	6	9.4	
T2	30	31.6	13	20.3	
T3	27	28.4	32	50	
T4	31	32.6	12	18.8	
Lymph node harvested					0.55
<12	25	25.3	14	21.2	
≥12	74	74.7	52	78.8	

*ASA, American Society of Anesthesiologists; CDmax, Maximum circumferential diameter; nRCT, Neoadjuvant radiotherapy and chemotherapy; SD, Standard deviation*.

The article "Safety and Feasibility of Robotic Natural Orifice Specimen Extraction Surgery in Colorectal Neoplasms During the Initial Learning Curve" was published in 2020. Journal: Front Oncol.

For Yao, in terms of gender, men and women accounted for 60.6% (60/99) and 39.4% (39/99), respectively. The mean age was 57.7 ± 12.8 years. The chief complaints were hematochezia (85.9%, 146/180), increased frequency of defecation (10.1%, 10/99), abdominal discomfort (2%, 2/99), and anal distention (2%, 2/99). The distance from the lower edge of the tumor to the anus was based on the colonoscopy report, with an average of 8.9 ± 3.7 cm, 4% (4/99) for <5 cm, 53.5% (53/99) for 5–10 cm, and 42.4% (42/99) for ≥ 10 cm. The proportion of patients who received neoadjuvant radiotherapy and chemotherapy was 17.2% (17/99). A total of 14 patients had abdominal or pelvic surgery history, accounting for 14.1%. ASA was classified as 4% (4/99), 47.4% (47/99), 47.4% (47/99), and 1% (1/99) in levels 1, 2, and 4. Cases for protective ileostomy accounted for 4% (4/99). A total of 93.9% (93/99) of histological types were tubular adenocarcinoma, 3 adenomas, 2 mucinous adenocarcinoma, and 1 neuroendocrine tumor. The average and the maximum CDmax (maximum circumferential diameter) of specimens were 3.5 ± 1.7 and 12 cm, respectively. The number of lymph nodes harvested ≥ 12 accounted for 74.7% (74/99), and the average number of lymph nodes harvested was 15 ± 5.1. According to the depth of tumor invasion, the T_is_, T1, T2, T3, and T4 stages were 0% (0/99), 7.4% (7/99), 31.6% (30/99), 28.4% (27/99), and 32.6% (31/99), respectively.

For Li, in terms of gender, men accounted for 66.7% (44/66) and women accounted for 33.3% (22/66). The mean age was 57 ± 13.2 years. The chief complaints were hematochezia (74.2%, 49/66), increased frequency of defecation (22.7%, 15/66), and routine examination (3%, 2/66). The distance from the lower edge of the tumor to the anus was based on the colonoscopy report with an average of 8.17 ± 3.18 cm, 10.6% (7/66) for <5 cm, 59.1% (39/66) for 5–10 cm, and 30.3% (20/66) for ≥ 10 cm. The proportion of patients who received neoadjuvant radiotherapy and chemotherapy was 7.6% (5/66). Ten patients had abdominal or pelvic surgery history, accounting for 15.2%. ASA was classified as 4.5% (3/66), 51.5% (34/66), 42.4% (28/66), and 1.5% (1/66) in levels 1, 2, and 4. Cases for protective ileostomy accounted for 3% (2/66). A total of 95.5% (63/66) of histological types were tubular adenocarcinoma, 2 adenomas, and 1 mucinous adenocarcinoma. The average and maximum CDmax of the specimen were 3.71 ± 1.43 and 7 cm, respectively. The number of lymph nodes harvested ≥ 12 accounted for 78.8% (52/66), and the average number of lymph nodes harvested for each case was 15 ± 4.7. According to the depth of tumor invasion, the T_is_, T1, T2, T3, and T4 stages were 1.6% (1/66), 9.4% (6/66), 20.3% (13/66), 50% (32/66), and 18.8% (12/66), respectively.

The article "Safety and Feasibility of Robotic Natural Orifice Specimen Extraction Surgery in Colorectal Neoplasms During the Initial Learning Curve" was published in 2020. Journal: Front Oncol.

### LC Analysis

The operation time of each case was recorded (Figures 2, 4). The LC was assessed via the CUSUM method. As the CUSUM_OT_ graph showed (Figures 3, 5), the peak point was observed at the 42nd and 15th cases for Yao and Li, respectively, after then, the operation time was decreased gradually. The beginning 42 and 15 robotic NOSES cases were considered as the initial LC for Yao and Li, respectively.

**Figure 2:** Graph of operative times plotted for each robotic NOSES for Prof. Yao.

**Figure 3:** Cumulative sum graph for operative time for Prof. Yao.

**Figure 4:** Graph of operative times plotted for each robotic NOSES for Prof. Li.

**Figure 5:** Cumulative sum graph for operative time for Prof. Li.

### Comparison of Safety and Feasibility Before and After the Completion of LC

The cases performed by Prof. Yao and Prof. Li can be divided into two parts (by the 42nd and 15th cases, respectively), in accordance with the completion of LC. The safety and feasibility of the two parts were compared (Table 2). For Yao, in terms of safety, only the operation time before the completion of LC (213.3 ± 67 min) was longer than after the completion of LC (143.8 ± 33.3 min). Other indices, such as postoperative hospital stay, intraoperative blood loss, conversion to laparotomy, incidence of anastomotic leakage, reoperation rate, and 90-day mortality rate had no significant statistical difference. In terms of feasibility, the dissected lymph node number, positive resection margin rate, and total cost between two parts had no significant statistical difference (*P* > 0.05). For Li, no significant statistical difference for all indices between two parts were observed (*P* > 0.05).

The article "Safety and Feasibility of Robotic Natural Orifice Specimen Extraction Surgery in Colorectal Neoplasms During the Initial Learning Curve" was published in 2020. Journal: Front Oncol.

**Table 2:** Comparision of safety and feasibility before and after LC completion.

	**Prof. Yao**			**Prof. Li**		
	**Before LC**	**After LC**	***P***	**Before LC**	**After LC**	***P***
**Safety**						
Operative time (min)	213.3 ± 67.0	143.8 ± 33.3	<0.01	266 ± 166.4	177.3 ± 39.3	0.59
Blood loss (ml)	50.5 ± 22.1	53 ± 19.1	0.547	44.7 ± 51	30.9 ± 26.7	0.328
Conversion to laparotomy (%)	0	0	N/A	0	0	N/A
Postoperative hospital stay (d)	10.1 ± 4.6	10.5 ± 9.1	0.785	14.5 ± 10.9	12.5 ± 6.6	0.396
Anastomotic leakage (n,%)	3/42, 7.14%	3/57, 5.3%	>0.99	1/15, 6.7%	1/51, 2%	0.938
Reoperation (n,%)	0/42, 0%	2/57, 3.5%	0.506	0/15, 0%	2/51, 3.9%	>0.99
90-day mortality (%)	0	0	N/A	0	0	N/A
**Feasibility**						
Lymph node harvested	15.4 ± 6.1	14.8 ± 4.2	0.598	14.4 ± 3.5	15.1 ±5	0.603
Positive resection margins (%)	0	0	N/A	0	0	N/A
Cost (CNY)	106,646 ± 14,364	114,956 ± 58,954	0.374	103,722 ± 12,429	103,696 ± 22,026	0.997

*LC, Learning curve; N/A, Not applicable; CNY, Chinese Yuan*.

## Discussion

The incidence of colorectal cancers per 100,000 population has decreased from 60.5 in 1976 to 46.4 in 2005 (5) and continued to decrease at a rate of ~2.9% per year or greater between 2005 and 2014 (6). In 2011, the reported incidence rate for colorectal cancer is 40.0 per 100,000 persons (7). In addition, mortality from colorectal cancer has decreased by almost 35% from 1990 to 2007 (8). The improvements in the incidence and mortality from colorectal cancer are thought to be a result of cancer prevention and early diagnoses through screening and improved treatment modalities. Nevertheless, colorectal cancer remains the fourth most frequently diagnosed cancer and the second leading cause of cancer death. In 2018, an estimated 43,030 new cases of rectal cancer will occur in the United States (25,920 cases in men, 17,110 cases in women) (6). Our study showed that the incidence for males, which is ~63% (104/165), is slightly higher than that for females and similar to that in the United States. Most of the patients complained of hematochezia and were administered and diagnosed by colonoscopy and biopsy. The sensitivity of the tumor markers was unsatisfactory. The sensitivity of the carcinoembryonic antigen was only 18.4% (28/152), whereas that of the carbohydrate antigens 242 and 199 were only 4.6% (7/152) and 5.7% (7/122), respectively.

Several randomized studies have identified that the conventional laparoscopic surgery for the treatment of patients with colorectal cancer has been maturing in recent years (9–13). Compared with open surgery, short-term endpoints with patients in the laparoscopic team show advantages, such as reduced blood loss and hospital stays and quick return of bowel function, but have prolonged operation times. No difference was seen in the completeness of resection and the percentage of patients with a positive circumferential resection margin, morbidity, or mortality. Moreover, the 3- and 5-year follow-up have shown no statistically significant difference in local recurrence, progression-free survival (PFS), or overall survival (OS) (9, 14). Many reports on laparoscopic NOSES for colorectal cancer are available (15–18), and this method has been proven to be safe and effective. In addition, numerous reports comparing laparoscopic NOSES with conventional laparoscopic surgery in colorectal surgery exist. Laparoscopic NOSES is safe and feasible with numerous advantages, including reduced pain and tissue trauma, fast recovery of intestinal function, and short postoperative hospital stay duration (19–23). Two meta-analyses involving 1,435 and 837 patients have also shown that compared with conventional laparoscopic surgery, NOSES may be a safe procedure that can significantly reduce the duration of hospital stay, accelerate postoperative recovery with improved cosmetic results, and in particular, minimize postoperative pain and complications while achieving similar oncological outcomes (24, 25). In June 2017, the China NOSES Alliance is established and released the *Expert consensus of natural orifice specimen extraction surgery in colorectal neoplasm (2017 edition)* to promote the application of NOSES (26). In addition, the International Alliance of NOSES issued the *International consensus on natural orifice specimen extraction surgery for colorectal cancer* in 2019 (27).

The article "Safety and Feasibility of Robotic Natural Orifice Specimen Extraction Surgery in Colorectal Neoplasms During the Initial Learning Curve" was published in 2020. Journal: Front Oncol.

The Da Vinci robot system has been approved by the FDA in 2000, and many reports of the robotic radical resection of colorectal cancer are available. However, in these reports, the specimens have been extracted through a small abdominal incision. Reports about robotic NOSES, particularly the retrospective analysis of small samples and case reports, are rare (28–31). According to our experience, especially in ultralow rectal cancer, robotic NOSES has advantages over laparoscopic NOSES. After all, the NOSES for colorectal neoplasm is a reconstruction surgery. No matter the reinforcement of the anastomosis or the suturing of the pelvic peritoneum, it needs to be sutured and knotted. Compared with conventional laparoscopic surgery, robotic surgery has more advantages in suturing and knotting, especially in a narrow pelvic cavity. Moreover, recent research shows robotics to have a faster LC in rectal cancer surgery than laparoscopy (32, 33).

In this study, the LC was assessed via the CUSUM method. Results showed that the estimated LC for robotic NOSES was achieved after the 42nd and 15th cases for Yao and Li, respectively. The LCs of the two surgeons were quite different. In our opinion, these differences can be ascribed to two reasons. First, the LC can be drastically different due to the different operative styles and experience of each surgeon. Shaw et al. have shown that the complex robotic colorectal surgery can be performed with reduced operative time and complications after 15 robotic cases (34). Foo et al. have shown that the LC for robotic-assisted total mesorectal excisions for a novice rectal surgeon is 25 cases (35). The data obtained by Jimenez et al. suggest that the estimated LC for robotic-assisted rectal cancer surgery is achieved after 21–23 cases (36). Park et al. have shown that the primary technical competence was achieved at the initial learning period of the 44th case in accordance with the robotic low anterior resection for rectal cancer (37). Second, Prof. Yao was the first surgeon to develop the robotic NOSES in our Department in March 2016, whereas Prof. Li started to develop robotic surgery in April 2017 with the support and guidance of Prof. Yao. Thus, the LC of Prof. Li can be shortened.

We also compared the outcomes of two surgeons before and after the completion of learning curve. The operation time of Yao before the completion of LC (213.3 ± 67 min) was longer than that after completion of LC (143.8 ± 33.3 min). The difference was statistically significant. Other indices in terms of safety, such as postoperative hospital stay, intraoperative blood loss, conversion to laparotomy, incidence of anastomotic leakage, reoperation rate, and 90-day mortality, had no significant statistical difference for Yao and Li. In terms of feasibility, the dissected lymph node number, positive resection margin rate, and total cost before and after the completion of LC lacked significant statistical difference (*P* > 0.05). Our study demonstrated that robotic NOSES in colorectal neoplasms is safe and feasible during the initial LC.

Our analysis has several limitations. First, the follow-up should be extended, and oncological outcomes, such as PFS and OS need to be verified. However, due to various reasons, many patients refused to return to hospital for adjuvant therapy or regular follow-up as our wishes. Insufficient compliance of patients leads to oncological outcomes could not be truthfully reflected. Second, this is a retrospective research. So, the integrity and accuracy of clinical data could not be guaranteed.

The article "Safety and Feasibility of Robotic Natural Orifice Specimen Extraction Surgery in Colorectal Neoplasms During the Initial Learning Curve" was published in 2020. Journal: Front Oncol.

## Conclusions

Cases before the completion of LC for robotic NOSES in colorectal neoplasms varied from 15 cases to 42 cases. Robotic NOSES is safe and feasible during the initial LC.

## Data Availability Statement

The raw data supporting the conclusions of this article will be made available by the authors, without undue reservation.

## Ethics Statement

The study was approved by the Ethics Committee of The Second Xiangya Hospital. The written informed consents of patients were been obtained.

## Author Contributions

HY: investigation, resources, writing-reviewing and editing, and supervision. TL, SL, and WC: investigation and resources. KL: methodology, software, and formal analysis. XJ: software and data curation. JZ: conceptualization, writing-original draft preparation, software, and data curation. All authors contributed to the article and approved the submitted version.

## Conflict of Interest

The authors declare that the research was conducted in the absence of any commercial or financial relationships that could be construed as a potential conflict of interest.
